# *In silico* analysis of regulatory networks underlines the role of miR-10b-5p and its target *BDNF* in huntington’s disease

**DOI:** 10.1186/2047-9158-3-17

**Published:** 2014-08-18

**Authors:** Sören Müller

**Affiliations:** 1 Molecular BioSciences, University of Frankfurt, Marie-Curie-Str.9, 60439 Frankfurt a.M., Germany

**Keywords:** Huntington, miRNA, Sequencing, Post-transcriptional regulation

## Abstract

Non-coding RNAs (ncRNAs) play various roles during central nervous system development. MicroRNAs (miRNAs) are a class of ncRNAs that exert their function together with argonaute proteins by post-transcriptional gene silencing of messenger RNAs (mRNAs). Several studies provide evidence for alterations in miRNA expression in patients with neurodegenerative diseases. Among these is huntington‘s disease (HD), a dominantly inherited fatal disorder characterized by deregulation of neuronal-specific mRNAs as well as miRNAs. Recently, next-generation sequencing (NGS) miRNA profiles from human HD and neurologically normal control brain tissues were reported. Five consistently upregulated miRNAs affect the expression of genes involved in neuronal differentiation, neurite outgrowth, cell death and survival. We re-analyzed the NGS data publicly available in array express and detected nineteen additional differentially expressed miRNAs. Subsequently, we connected these miRNAs to genes implicated in HD development and network analysis pointed to miRNA-mediated downregulation of twenty-two genes with roles in the pathogenesis as well as treatment of the disease. *In silico* prediction and reporter systems prove that levels of *BDNF*, a central node in the miRNA-mRNA regulatory network, can be post-transcriptionally controlled by upregulated miR-10b-5p and miR-30a-5p. Reduced *BDNF* expression is associated with neuronal dysfunction and death in HD. Moreover, the 3’UTR of *CREB1* harbors a predicted binding site for these two miRNAs. *CREB1* is similarly downregulated in HD and overexpression decreased susceptibility to 3-nitropropionic-induced toxicity in a cell model. In contradiction to these observations, it is presumed that miR-10b-5p upregulation in HD exerts a neuroprotective role in response to the mutation in the huntingtin gene. Therefore, the function of miR-10b-5p and especially its effect on *BDNF* expression in HD requires further academic research.

## Introduction

Huntington’s disease (HD) is a fatal hereditary neurodegenerative disorder characterized by unwanted choreatic movements, behavioral manifestations and dementia [1]. In the caucasian population HD appears with an incidence of one per 10,000-20,000 per year in middle age (30-50 years) [2]. The disease is caused by a genetic disorder. An elongation of the CAG trinucleotide repeat (36 repeats or more) is observed within the coding region of the huntingtin (*HTT*) gene [3]. This mutation yields a protein with deleterious functions for brain cells and even impairs the ability of normal HTT to exert fundamental molecular activities in the neurons [4]. As a consequence, neurons predominantly degenerate in the brains of affected patients [4]. While the altered biological processes finally leading to neurodegeneration remain poorly understood, changes in messenger RNA (mRNA) expression point to transcriptional dysregulation as a central mechanism [5]. Beside deregulation of mRNAs, also differential expression of microRNAs (miRNAs) has been linked to HD [6]. MiRNAs are a class of small non-coding RNAs (sncRNAs) that can repress gene expression through translational repression or mRNA deadenylation and decay by base pairing to partially complementary sites [7]. Recent research has examined the role of miRNAs in HD using next generation sequencing (NGS) and identified between five and 85 deregulated miRNAs [8,9]. Hoss and colleagues [9] related five upregulated miRNAs (miR-10b-5p, miR-196a-5p, miR-196b-5p, miR-615-3p and miR-1247-5p) located in the HOX gene cluster to HD pathogenesis. Nevertheless, target and differential expression analysis with strict parameters revealed only one validated, downregulated target gene (*KRT5*) of these miRNAs. Therefore, their function in HD pathogenesis mostly remains unclear.

In order to shed light on the consequences of miRNA deregulation in HD we used omiRas [10] to re-analyze the dataset of Hoss and co-workers consisting of small RNA-Sequencing (sRNA-Seq) libraries derived from twelve HD and nine unaffected control brain tissue samples in FASTQ format. In extension to the five miRNAs identified by Hoss and colleagues we detected nineteen additional miRNAs as differentially expressed. Furthermore, we assigned functions to differentially expressed miRNAs via the interaction tool of omiRas. Analysis revealed *BDNF* as a validated target of two upregulated miRNAs (miR-10b and miR-30a), *CREB1* is predicted to be post-transcriptionally controled by the same two miRNAs. The potential miRNA-mediated downregulation of several major player genes in HD pathogenesis underlines the feasibility of miRNAs as therapeutic targets in HD.

## Materials and methods

### Dataset collection and preprocessing

A publicly available sRNA-Seq expression dataset of twelve HD and nine control brain samples from the prefrontal cortex was downloaded from Array Express (E-MTAB-2206) in FASTQ format. The 3’ sequencing adapter (TCGTATGCCGTCTTCTGCTTGAAA) was removed from the reads with cutadapt [11]. Subsequently, low quality stretches below a SANGER quality score of 20 were additionally trimmed from each end of the reads (-q 20). Only reads with a minimum length of fifteen base pairs after clipping were used for further analysis(-m 15). A list of differentially regulated genes identified in Microarray data of sixteen HD patients’ prefrontal cortex and fifteen controls cases published by Hodges and co-workers [5] was retrieved in XLS format and intersected with a list of genes with implication in HD, as defined by the HD crossroads database [12].

### MiRNA quantification, differential expression and target analysis

Samples were uploaded to omiRas and analyzed as described previously [10]. In contrast to Hoss and colleagues we tested for differential expression in “gene-est-only” mode of DESeq [13], which is recommended if more than seven replicates per condition are available. MRNA targets with involvement in HD pathogenesis (see dataset collection) of differentially expressed miRNAs were identified with the “interactive network tool” of omiRas. An interaction between a miRNA and a coding-gene is assumed to be valid if the following two criteria apply: (a) Three or more of seven miRNA-mRNA interaction databases support the interaction. (b) The expression of the miRNA/mRNA pair is inverse. The miRNA is significantly downregulated and the mRNA is upregulated or *vice versa*. Interactions between gene products of deregulated genes were detected *via* STRING database.

## Results

The results for the comparison of twelve HD and nine control brain samples is available from omiRas (http://tools.genxpro.net/omiras/10eea4eb58d1/results/). Our analysis confirms the upregulation of miR-10b-5p, miR-196a-5p, miR-196b-5p, miR-615-3p and miR-1247-5p in HD. In addition, we detect nineteen other differentially expressed miRNAs, of which four are down- and fifteen upregulated. The expression values in both conditions as well as the corrected p-value for each miRNA are given in Table 1. The lower number of differentially expressed miRNAs in comparison to previous studies [8,14] can be explained by the elimination of false positive candidates due to a reliable estimation of biological variance. The interaction network in Figure 1 comprises 65 protein products of downregulated genes with 121 protein-protein interactions. Hubs in the network represented by nodes with the most protein-protein interactions are Calmodulin 1 (*CALM1*) with twelve interactions and brain-derived neurotrophic factor (*BDNF*) with nine interactions. The downregulation of mRNAs coding for the proteins in the network is potentially caused by eight miRNAs with predicted binding sites in their 3’UTR. Approximately one third (22) of all mRNAs are predicted targets of miRNAs, four genes can be post-transcriptionally controlled by more than one miRNA (*BDNF*, *CALM1*, *CNR1*, *CREB1*). The hub genes *BDNF* and *CALM1* harbor a binding site for miR-10b-5p, 196a-5p, 196b-5p and 30a-5p in their 3’UTR. *CREB1* and *BDNF* are predicted targets of miR-10b and miR-30a, whereas the regulation of *BDNF* has recently been experimentally verified in the prefrontal cortex [15,16].

**Table 1:** Deregulated miRNAs in HD

**miRNA**	**NEV Control**	**NEV HD**	**foldChange**	**FDR**	**Other studies**
miR-196a-5p	0.00	19.01	Inf	1.4E-010	[9,14]
miR-891a	48.39	101.39	2.10	0.00001	-
miR-10b-5p	1011.52	30689.38	30.34	0.00003	[9]
miR-4645-3p	3.66	9.44	2.58	0.0001	-
miR-1247-5p	135.61	309.04	2.28	0.0004	[9]
miR-10b-3p	0.00	5.28	Inf	0.0026	-
miR-363-3p	2239.63	3274.71	1.46	0.0033	[8]
miR-30a-3p	5223.90	6943.31	1.33	0.0048	[8]
miR-125b-2-3p	17177.77	20740.93	1.21	0.0052	-
miR-615-3p	0.00	5.45	Inf	0.0065	[9]
miR-196b-5p	1.09	10.17	9.33	0.0134	[9]
miR-127-3p	175251.70	224611.39	1.28	0.0194	-
miR-208b	75.76	112.90	1.49	0.0217	-
miR-302a-5p	2.67	6.93	2.60	0.0451	-
miR-2682-5p	212.76	299.86	1.41	0.0451	-
miR-30a-5p	171969.53	228298.92	1.33	0.0451	[8]
miR-770-5p	333.36	445.55	1.34	0.0451	-
miR-130a-3p	4740.57	6385.28	1.35	0.0451	-
miR-92b-5p	40.62	57.17	1.41	0.0451	-
miR-449a	20.31	32.65	1.61	0.0451	-
miR-3139	8.59	2.27	0.26	0.0031	-
miR-4449	10.95	2.75	0.25	0.0163	-
miR-4521	335.51	168.04	0.50	0.0194	-
miR-138-2-3p	94.11	74.60	0.79	0.0194	-

MiRNAs upregulated in HD brains are indicated by a fold-change ***>***1, downregulated miRNAs by a fold-change ***<***1. NEV corresponds to the normalized expression value and FDR is the corrected p-value. Other studies indicates if any study different from this has likewise reported the miRNA deregulation in HD.

**Figure 1:** **MiRNA-mRNA interaction network in HD.** Downregulated genes/gene products with implication in HD pathogenesis are represented by red circles. Interactions between proteins are visualized with blue lines, predicted post-transcriptional regulation of mRNAs by miRNAs is indicated by a dotted grey line.

## Discussion

We extend the report of Hoss and co-workers based on NGS miRNA expression profiles of twelve HD and nine healthy control brain samples. Re-analysis of the dataset reveals 24 differentially expressed miRNAs in HD, 20 of these up- and four downregulated. Regulatory network analysis comprising genes involved in HD pathogenesis with decreased expression underlines the role of the most significantly upregulated miRNA, miR-10b-5p, that targets *BDNF* and *CREB1*.

BDNF is a secreted neurotrophic factor, which represent a class of molecules that contribute essentially to the survival of the peripheral and central nervous system, and reduced level of *BDNF* mRNA as well as protein have been found in HD cerebral cortex and striatum [17]. BDNF is required in striatal neurons for survival and activity. The largest proportion of striatal BDNF is initially produced in the frontal cortex and subsequently transported to the striatum [18]. YAC 128 mice that were transplanted with BDNF overexpressing MSCs in the striatum show a significantly reduced amount of neuronal loss [19]. Downregulation of *BDNF* has been directly associated with the mutation of wild-type *HTT*[17]. Our analysis extends the regulatory mechanism leading to *BDNF* downregulation in HD to miR-10b-5p and 30a-5p which are significantly upregulated in HD and have been shown to target the 3’UTR of the *BDNF* transcript [15,16]. Upregulation of *BDNF* levels in the striatum/cortex are a potential therapeutic strategy in HD treatment [18] and our analysis points to an inhibition of miRNAs by antagomiRs to achieve this goal. Mir-10b antagomirs have *inter alias* been used for therapeutic silencing of miR-10b to inhibit metastasis in a mouse mammary tumor model [20]. In contradiction to these observations, miR-10b-5p expression enhanced the survival of PC12 Q73 cells and its upregulation in HD may be a neuroprotective response to the HTT mutation [9]. Therefore, the role of miR-10b-5p and especially its effect on *BDNF* expression in HD requires further academic research.

*CREB1* encodes a transcription factor that is a member of the leucine zipper family of DNA binding proteins. CREB1 induces transcription of genes in response to hormonal stimulation of the cAMP pathway. Members of the CREB family are essential for the maintenance of cell viability in various tissues and stages of development [21]. Reduced *CREB1* expression has been reported in HD and mutant Htt represses *CREB1* expression by a direct interaction with the CREB-binding protein [22]. Lack of CREB1 expression during development of the central nervous system leads to substantial apoptosis of postmitotic neurons [21]. The CREB signaling pathway has been suggested for pharmacological intervention in neurodegenerative disorders like HD [21]. The 3’UTR of *CREB1* harbors predicted binding sites of miR-10b-5p, 30a-5p and 196a-5p, which makes antagomiRs a potential approach for intervention in CREB signalling. Nevertheless, these interactions lack experimental validation and form a basis for further research.

Taken together our analysis underlines the role of miRNAs in HD pathogenesis. The regulatory network of deregulated genes and miRNAs may now spur further research in the field of HD. We provide a set of miRNA-mRNA interactions that currently lack experimental validation and point to miRNAs that are potential targets for treatment with antagomiRs. The validity of the predicted interactions between downregulated genes and upregulated miRNAs is underlined by the recent validation of four interactions in the network (miR-10b-5p-*BDNF*, miR-30a-5p-*BDNF*, miR-30a-5p-*AP2A1*, miR-30a-5p-*PPP3CA*[23]).

## Competing interests

The author declares that they have no competing interests.
